# Cohort Study Summary of the Effects of Carboprost Tromethamine Combined with Oxytocin on Infant Outcome, Postpartum Hemorrhage and Uterine Involution of Parturients Undergoing Cesarean Section

**DOI:** 10.1155/2022/2233138

**Published:** 2022-08-25

**Authors:** Xiaoyan Gong, Xiaohui Wu

**Affiliations:** Department of Obstetrics and Gynecology, Yiwu Fuyuan Private Hospital, China

## Abstract

**Background:**

Carboprost tromethamine injection has a high safety factor in clinical application and has a good effect on uterine smooth muscle and vasoconstriction. Carboprost aminobutyriol combined with oxytocin may be beneficial to infant outcome and uterine involution after cesarean section.

**Objective:**

To investigate the effects of carboprost tromethamine combined with oxytocin on infant outcome, postpartum hemorrhage, and uterine involution in parturients undergoing cesarean section.

**Methods:**

A total of 120 parturients undergone cesarean section in our hospital from February 2019 to April 2021 were selected as the object of study. The parturients were randomly divided into control group (*n* = 60) and research group (*n* = 60). The control group was treated with oxytocin, and the research group was treated with carboprost aminobutyriol combined with oxytocin. The amount of maternal bleeding, uterine floor decline index, the end of lochia, poor rate of uterine involution, infant outcome, and the incidence of adverse drug reactions were compared between the two groups.

**Results:**

The amount of bleeding in the research group was significantly lower than that in the control group (*P* < 0.05). The position of the last uterine floor and the index of uterine floor downward movement in the research group were significantly higher than those in the control group (*P* < 0.05). The disappearance time of bloody lochia and serous lochia in the research group was significantly shorter than that in the control group (*P* < 0.05). The end time of lochia in the research group was higher than that in the control group, and the rate of uterine involution in the research group was lower than that in the control group (*P* < 0.05). The neonatal weight and Apgar score in the research group were higher than those in the control group, and the hospitalization rate of neonatal ICU in the research group was significantly lower than that in the control group. The incidence of adverse reactions in the research group was significantly lower than that in the control group (*P* < 0.05).

**Conclusion:**

Carboprost aminobutyriol combined with carbestatin can effectively prevent the occurrence of bleeding after cesarean section, improve uterine involution, and improve neonatal birth quality, which is worth popularizing.

## 1. Introduction

Under the influence of traditional concepts and customs, the cesarean section rate has been increasing year by year [1]. In 2014, the “Chinese Journal of Obstetrics and Gynecology” reported that the cesarean section rate in China has now reached 54%. The uterine birth rate is even as high as 72% [2]. The risk of postpartum hemorrhage and uterine involution is greatly increased. Some patients will be accompanied by adverse infant outcomes, so it is necessary to choose targeted drugs for prevention [3, 4].

Among the factors causing postpartum hemorrhage, uterine weakness accounts for 90% [5]. At present, oxytocin is the first choice for the prevention and treatment of postpartum uterine weakness [6–8]. It has the characteristics of quick effect, obvious effect of promoting uterine contraction, and short half-life, so it has been widely used in clinical treatment. Oxytocin can selectively bind to the corresponding receptors in uterine smooth muscle cells and increase the flow of calcium ions inside and outside the cells, thus promoting the contraction of uterine smooth muscle [9, 10]. However, when it is used in large doses, it can cause hypertension or water retention [11].

Carboprost tromethamine (CTI) is a PG-F2*α* derivative (15-methyl PGF2a). The main active ingredient is carboprost tromethamine. The half-life is longer than other uterine contraction drugs, enhancing the utilization of biological activity, and reducing the adverse reactions of the drug [12]. Carboprost tromethamine injection has a high safety factor in clinical application. Because PG is widely distributed in human tissues, it plays a good role in uterine smooth muscle and vasoconstriction. It is able to take effect quickly after intramuscular injection and further enhances the contractile effect of uterine smooth muscle by increasing the amplitude and frequency of uterine contraction [13, 14]. Based on this, this study focuses on the effects of carboprost tromethamine combined with oxytocin on infant outcome, postpartum hemorrhage, and uterine involution after cesarean section.

## 2. Materials and Methods

### 2.1. General Information

A total of 120 parturients undergoing cesarean section in our hospital from February 2019 to April 2021 were selected as the object of study. The parturients were randomly divided into control group (*n* = 60) and research group (*n* = 60). The control group was treated with oxytocin, and the research group was treated with carboprost tromethamine combined with oxytocin. In the control group, the age was 21-44 years old, with an average of 32.91 ± 2.55 years, and in the research group, the age was 20-45 years old, with an average age of 32.67 ± 2.58 years. This study was a double blind test. This study was approved by the Ethics Committee in our hospital.

Selection criteria are as follows: (1) parturients undergoing cesarean section, newborn weight ≥2500 g, <4000 g; (2) there were no serious complications during prenatal examination; and (3) the incision of cesarean section was transverse.

Exclusion criteria are as follows: (1) infection, ulceration, and other skin lesions in the treatment area; (2) longitudinal incision; (3) postoperative heart failure, pulmonary edema, and other serious complications; (4) massive bleeding during and after operation, that is, the amount of bleeding is greater than 1000 ml, uterine B-Lynch suture, uterine cavity packing, etc.; (5) those who could not touch the floor of the uterus clearly because of thick abdominal fat; (6) those with tuberculosis, syphilis, AIDS and other infectious diseases; (7) those with single or multiple uterine leiomyomas larger than 5 cm, those who underwent Hyster myomectomy during the operation, patients with adenomyosis, etc.; (8) those who underwent the third or more cesarean section; and (9) those with unstable systemic diseases and could not be tolerated.

Elimination standards are as follows: (1) those who were unable to complete the course of treatment for some reason; (2) those who needed to drop out in the course of treatment because of adverse reactions; (3) those who accepted other parturients who affect the treatment of this study at the same time during treatment or follow-up; and (4) those who needed to be excluded for other reasons.

### 2.2. Methods

In the control group, 20 U of oxytocin (manufacturer: Henan Furen Huaiqingtang Pharmaceutical Co., Ltd.; approval number: H19993526) was injected into the uterine body muscle after delivery. 10 U of oxytocin was injected intravenously at the same time. On this basis, the research group was directly injected with carboprost tromethamine injection (manufacturer: Fama West Puqiang Pharmaceutical Co., Ltd., imported drug registration number: H20120388) 0.25 mg.

### 2.3. Observation Index

#### 2.3.1. Postpartum Hemorrhage Volume

Gauze weighing method is used to measure the amount of hemorrhage volume. The intraoperative bleeding time, 2 hours postpartum bleeding volume, and 24 hours postpartum hemorrhage in the two groups were observed and recorded.

#### 2.3.2. Uterine Fundus Decline Index

The descending height of the uterine floor: the descending height of the uterine floor was measured at the same time every day (8-9 am). The patient was told to lie flat on the treatment bed after emptying the bladder. The descending height of the uterine floor (cm) = the first measurement of uterine length (cm) − the last measurement of uterine length (cm). Fundus decline index = (first measurement of uterine length − last measurement of uterine length)/(first measurement of uterine length) × 100%.

#### 2.3.3. Defective Rate of Involution of Uterus

Lochia mainly record the time when bloody lochia and serous lochia are completely clean and those whose lochia is not completely clean 42 days after operation.

#### 2.3.4. Defective Rate of Involution of Uterus

Bad rate of uterine involution: rate of bad involution = (number of people with lochia for more than 42 days)/(total number of people) × 100%.

#### 2.3.5. Infant Outcome

The infant outcomes of the two groups were counted.

#### 2.3.6. Incidence of Adverse Reactions

The incidences of chest tightness, dizziness and headache, abdominal discomfort, facial flushing, nausea, and vomiting were calculated between the two groups.

### 2.4. Statistical Analysis

SPSS23.0 statistical software was adopted to process the data. The measurement data were presented as ($\bar{x}\pm \text{s}$). The group design *t*-test was adopted for the comparison, and the analysis of variance was adopted for the comparison between multiple groups. Dunnett's test was adopted for comparison with the control group. The counting data were presented in the number of cases and the percentage. *χ*2 test and multiple Logistic regression were adopted to analyze the risk factors related to the prognosis of children. The difference exhibited statistically significant, and the difference was statistically significant (*P* < 0.05).

## 3. Results

### 3.1. Comparison of the Amount of Maternal Bleeding

The amount of blood loss during operation, 2 hours after operation, 24 hours after operation, and total blood loss in the research group were significantly lower than those in the control group (*P* < 0.05, Table 1).

### 3.2. Total Amount of Bleeding

There was no significant difference in the initial position of uterine floor between the two groups (*P* > 0.05). The position of the last uterine floor in the research group was lower than that in the control group, and the uterine floor decline index in the research group was higher than that in the control group, and the difference was statistically significant (*P* < 0.05, Table 2).

### 3.3. Comparison of the End of Lochia

The end time of bloody lochia and serous lochia in the research group were shorter than those in the control group, and there are statistically significant differences between groups (*P* < 0.05, Table 3).

### 3.4. Comparison of Defective Rate of Involution of Uterus

The 42-day end of lochia in the research group was higher than that in the control group. The rate of poor uterine involution was statistically significantly lower than that in the control group, and there are statistically significant differences between groups (*P* < 0.05, Figure 1).

### 3.5. Comparison of Infant Outcomes

The neonatal body weight and neonatal Apgar score in the research group were higher than those in the control group. The neonatal admission rate in the ICU was lower than that in the control group, and there are statistically significant differences between groups (*P* < 0.05, Table 4).

### 3.6. Comparison of the Incidence of Adverse Reactions

The incidences of chest tightness, dizziness and headache, abdominal discomfort, facial flushing, nausea, and vomiting in the research group were significantly lower than those in the control group, and there are statistically significant differences between groups (*P* < 0.05, Figure 2).

## 4. Discussion

Cesarean section is an important operation in the field of obstetrics [15]. The cesarean delivery has basically replaced vaginal midwifery operations such as mid-to-high forceps and breech traction, which are more damaging to the fetus [16]. Cesarean section has become an effective means to solve dystocia and some obstetrical complications and save the lives of parturients and perinatal infants [17]. However, the maternal mortality and perinatal mortality will not continue to decrease with the unlimited increase of the cesarean section rate. A domestic study showed that the cesarean section rate was approximately 19.5% in 1980-1984 and rose to approximately 25.4% in 1985-1988 [18, 19]. In China, according to the national symposium on cesarean section in 1989, the rate of cesarean section was only 1% or 2% in the 1950s, rising to 22% in 1988 [20]. Since the 1990s, the rate of cesarean section has risen sharply, and the rate of cesarean section in Shanghai has reached 45.9%. And some hospitals are more than 60.0%, or even 80.0% [21]. At present, it has not reached a stable level [22]. Compared with vaginal delivery, cesarean section is a transabdominal incision to remove the fetus. The incidence of intraoperative bleeding, postoperative thrombosis, placenta previa, and uterine rupture in cesarean section is much higher than that in vaginal delivery. Therefore, taking targeted treatment measures to prevent postpartum hemorrhage and reduce the incidence of uterine involution has important clinical value [23–25].

Postpartum hemorrhage (PPH) is a type of disease in which the amount of blood loss exceeds 500 ml within 24 hours after vaginal delivery and exceeds 1000 ml during cesarean section. It is the leading cause of maternal death in China, accounting for 40.5% of maternal mortality [26–28]. PPH develops rapidly and critically. Massive hemorrhage in a short period of time can cause hemorrhagic anemia, hemorrhagic shock, multiple organ failure, and even more serious life-threatening maternal life [29, 30]. Therefore, postpartum hemorrhage has a significant impact on the prognosis of pregnant women and it affects the process of uterine recovery. The process of uterine recovery mainly depends on the spontaneous contraction of uterine muscles and the regeneration of endometrium, which generally takes about 6 weeks [31]. On the other hand, if the uterus has not recovered to the nonpregnant state after more than 6 weeks, it is the poor involution of the uterus. In the process of uterine involution, many reasons may lead to postpartum uterine involution, especially that uterine weakness is the most common [32]. The most common clinical symptoms of uterine involution in uterine atony type were continuous or slow decline of uterine floor, excessive vaginal bleeding, and prolonged bleeding time. Colorful ultrasound examination showed that the anterior and posterior diameter of uterus was significantly larger than the normal value [33]. The key point for the prevention and treatment of postpartum uterine involution is how to promote postpartum uterine contraction, reduce postpartum hemorrhage, and reduce lochia time [34–37].

After long-term clinical practice, there are many methods for the treatment of uterine atony PPH, including surgical hemostasis and drug therapy. The surgical hemostasis includes uterine artery ligation, arterial embolization, and uterine compression suture. However, for postpartum hemorrhage caused by uterine weakness, placental abnormality, uterine rupture, and abnormal blood coagulation, hysterectomy should be directly selected when conservative treatment is ineffective [38–40]. Traditional drug therapy, such as kabetosin and ergoxin, has great limitations. Among which, oxytocin has a short half-life, rapid drug metabolism, and short-term effect on uterine smooth muscle, while ergoxin can only contract the upper segment of uterus. The adverse drug reactions are serious, which can affect the patient's blood pressure, resulting in the decrease of plasma osmotic pressure and the increase of circulatory blood volume [41–43]. Prostaglandin, represented by carboprost tromethamine (CTI), can stimulate blood vessels, bronchi, uterus, and smooth muscle and especially promote uterine contraction, so it has been widely used in the treatment of uterine atony PPH and achieved ideal clinical effect [44].

Prostaglandins are a kind of physiologically active derivatives of unsaturated fatty acids, which not only stimulate the bronchi, gastrointestinal smooth muscle, uterus, and blood vessels, but also cause them to contract. Prostaglandins bind to specific receptors and constantly affect blood and related cells in mediating cell proliferation, differentiation, apoptosis, and other activities. It plays a role in the regulation of female reproductive function and the balance of the cardiovascular system during childbirth [45–47]. CTI is a prostaglandin injection that contains (15 s)-15 methyl derivatives of natural prostaglandin F2 *α*. It has a strong contractile effect on the uterus at all stages of pregnancy. CTI can induce rhythmic uterine contraction by binding to oxytocin receptors on uterine smooth muscle [48]. Under normal circumstances, the level of oxytocin receptor in uterine smooth muscle is low. With the increase of pregnancy time, the level of oxytocin receptor in uterine smooth muscle increases gradually and reaches its peak during delivery [49]. On the other hand, it can increase the intrauterine pressure and the tension of uterine smooth muscle, resulting in a natural, efficient, and thorough hemostatic effect [50]. As a new type of prostaglandin, CTI is not only widely used in clinic, but also has strong efficacy. CTI is the carrier of calcium ions. It will activate acrosin, regulate the activity of cyclic adenylate, promote cell division and differentiation, and shorten the process of labor. CTI can effectively control adenylate cyclase, produce catalysis, and promote cell maturation as well [51]. CTI has a long and lasting irritating effect on uterine smooth muscle [52]. At the same time, CTI also has strong biological activity, which can promote platelet coagulation, thus shorten the process of blood coagulation, and stop bleeding in a short time. Therefore, compared with other prostaglandins, CTI is effective with fewer adverse reactions and stronger hemostatic effect [53].

It is proved that CTI plus oxytocin is more efficiently in the therapies of postpartum hemorrhage. This is mainly due to the short half-life (3~4min) and rapid metabolism of Cabe oxytocin, which cannot continuously stimulate the intrauterine smooth muscle of pregnant women. Substituting methyl group for 15-hydroxyl group in CTI can not only prolong the half-life and enhance the biological activity, but also continue to contract the uterus. 34 patients with postpartum hemorrhage were ineffective in basic treatment were included [54]. After injection of CTI combined with oxytocin, the average amount of bleeding was much lower than that of patients who did not take this measure. In the other study, the total effective rate of CTI combined with oxytocin in the treatment of postpartum hemorrhage was 95%, which was significantly higher than that of oxytocin combined with uterine massage [55, 56]. In addition, except for the short half-life of oxytocin, the dosage of oxytocin is also limited [57]. CTI has long half-life, long-lasting efficacy, and strong biological activity. In combination with oxytocin, it can increase the level of calcium ions in the maternal cytoplasm and enhances the contractility of the uterine muscle fibers. It is effective in stimulating contraction of uterine smooth muscle within 24 hours after delivery to control bleeding and improve the efficacy of the treatment [58, 59]. This study still has some shortcomings. Firstly, the quality of this study is limited due to the small sample size we included in the study. Secondly, this research is a single-center study, and our findings are subject to some degree of bias. Therefore, our results may differ from those of large-scale multicenter studies from other academic institutes. This research is still clinically significant, and further in-depth investigations will be carried out in the future.

To sum up, compared with the treatment with oxytocin alone, carboprost tromethamine combined with oxytocin can effectively prevent the occurrence of postpartum hemorrhage after cesarean section. The uterine involution and the birth quality of newborns can be improved with fewer adverse drug reactions. Therefore, it is worthy of clinical application.

## Figures and Tables

**Figure 1:** Comparison of defective rate of involution of uterus.

**Figure 2:** Comparison of the incidence of adverse reactions.

**Table 1:** Comparison of the amount of postpartum hemorrhage between the two groups ($\bar{x}\pm \text{s}$, ml).

Group	*N*	Intraoperative bleeding volume	Amount of blood loss 2 hours after operation	Blood loss 24 hours after operation	Total amount of bleeding
Control group	60	546.93 ± 83.52	87.94 ± 38.42	204.91 ± 83.75	725.92 ± 86.42
Research group	60	454.95 ± 79.34	74.29 ± 16.29	173.85 ± 84.33	638.94 ± 103.95
*t*		6.184	2.533	2.024	4.983
*P*		<0.05	<0.05	<0.05	<0.05

**Table 2:** The uterine fundus decline index between the two groups ($\bar{x}\pm \text{s}$).

Group	*N*	Initial position of uterine floor (cm)	The position of the last uterine floor (cm)	Uterine fundus decline index (%)
Control group	60	19.84 ± 1.44	16.79 ± 2.44	15.49 ± 2.44
Research group	60	19.89 ± 1.55	15.45 ± 0.45	16.31 ± 2.31
*t*		0.183	4.183	2.333
*P*		>0.05	<0.05	<0.05

**Table 3:** The end of lochia between the two groups ($\bar{x}\pm \text{s}$, d).

Group	*N*	End time of bloody lochia (d)	End time of serous lochia (d)
Control group	60	9.38 ± 2.11	22.49 ± 6.42
Research group	60	8.01 ± 2.21	17.29 ± 7.33
*t*		3.473	4.133
*P*		<0.05	<0.05

**Table 4:** The infant outcomes between the two groups ($\bar{x}$±s).

Group	*N*	Newborn weight (kg)	Apgar score of newborns	Newborn in ICU
Control group	60	3021.44 ± 133.44	9.21 ± 0.31	17 (28.33)
Research group	60	3253.81 ± 233.22	9.83 ± 0.01	1 (1.67%)
*t*/*χ*2		6.698	15.483	16.732
*P*		<0.05	<0.05	<0.05

## Data Availability

No data were used to support this study.
